# A Design Model of Music Teaching and Auxiliary System Based on Artificial Neural Networks

This article has been retracted.

**DOI:** 10.1155/2022/4580027

**Published:** 2022-08-16

**Authors:** Bo Chen

**Affiliations:** Hunan International Economics University, ChangSha 410205, China

## Abstract

The Internet has now ingrained itself into every aspect of people's lives and has grown to be a necessity. Machine learning technology is applied to the design of music teaching and teaching assistant systems with the aim of bringing convenience to students and teachers in teaching and learning and improving teaching efficiency and quality through the design and implementation of a friendly and interactive intelligent music assistant teaching system. The B/S mode framework aids in the realisation of the hierarchy and module structure of the system design during the system implementation process. Last but not least, this paper looks at the system modules, confirms all of the system's operations, and makes sure each functional module is working properly. The algorithm is straightforward, effective, simple to use, and user-friendly, and the system is expandable, portable, and transparent. It is an excellent teaching tool for music.

## 1. Introduction

The computer has demonstrated significant advantages in information storage, presentation, and calculation and has established itself as a necessary tool for modern work, study, and daily life [1]. Computer-aided systems are becoming more prevalent and playing a significant role in all spheres of life as a result of the ongoing innovation and development of computers and AI (artificial intelligence). The term “computer-aided system” is a general one that refers to systems that use computers to help with various tasks across many industries [2]. We are unable to function without the assistance of computer-aided systems in both daily life and military operations. The use of computer-aided systems in education is growing daily and has a significant impact. As a learning tool for the human reasoning model in other areas of instruction, CAI is also increasingly practical [3]. The primary goal of the computer-assisted teaching system known as CAI (computer assisted instruction) is to give teachers and students access to convenient teaching techniques. The interface between a teaching system, subject matter experts, knowledge engineers, and general users is called a man-machine interface (HMI). Data, information, commands, output, and information display are all done using it. The use of high technology, such as multimedia, AI, databases, and remote networks, has replaced the traditional educational model of using blackboards, books, and teaching materials [4]. The intelligent teaching system in colleges and universities, which is closely related to the modernization of teaching, has gradually incorporated CAI. A comprehensive, effective, and diversified music teaching mode within the network information environment is built through the research and development of music teaching assistant systems. By utilising the Internet's rapid information dissemination, wealth of resources, and lack of geographic restrictions, we can effectively and conveniently assist students in learning, completing, and expanding their musical knowledge.

This CAI-dependent education mode can increase students' interest, improve teachers' education levels, and improve teaching quality. Now, more and more schools have applied CAI, and the effect is remarkable [5, 6]. It can not only realize the effectiveness of the music teaching system, but also realize online music knowledge imparting, students' study situation investigation, assessment and performance analysis, and organic interaction between teachers and students [7]. Thereby providing an interactive system for teachers and students, and prompting students to learn music curriculum knowledge easily and happily; and teachers can fully understand the actual needs of students. At present, there are many intelligent network-based teaching assistant systems at home and abroad, but the degree of intelligence is not high. Compared with mastering the learning situation of each student, a great task for teachers is to know the knowledge of a group of students rather than just one student [8]. The existing CAI system faces many challenges, which mainly have the following four problems: (1) Lack of openness and human-computer interaction ability. (2) Ignoring the characteristics of the course itself, the limitation of fixed content makes the application of courseware narrow. (3) Teaching is not targeted and lacks intelligence. (4) Lack of timeliness leads to a lack of interaction between teachers and students. This paper introduces machine learning technology to create a music teaching assistant system in accordance with the actual circumstances of contemporary music instruction. The following are the innovations of this paper:

1. This paper designs and builds a music teaching assistant system in response to the issues with digital music classroom instruction and the shortcomings of conventional CAI. This system not only pays attention to the learning of the students but also pays attention to the assessment of the students' learning environment. To better realise the goal of assisting teaching, combine systematic teaching evaluation with independent learning. This will increase contact and interaction between teachers and students. For pertinent researchers, this serves as a reference and a direction.
2. This paper determines the functions of the system to be developed, the mode of system architecture, and the modules of the system by analysing the actual needs of music theory, common sense, and appreciation teaching. The data persistence layer and presentation layer of the system are realised during system implementation with the aid of the ThinkPHP software framework and its features. According to the research, this system can handle a lot of data interaction and has real-time and security features.

The goal of this paper is to design and implement a system to assist music teachers. The article is divided into five chapters with the following specific organisation: The introduction is the first chapter. This section primarily covers the research background, research objectives, significance, inventiveness, and organisational structure of this study. A review of the literature is covered in the second chapter. This chapter provides the research concepts for this paper as well as a summary of the current state of domestic and international research and application. The third chapter is split into two sections. The related technologies of machine learning are discussed, examined, and a summary of the relevant CAI contents is provided in Section 3.1. A machine learning-based music teaching assistant system is built in Section 3.2, and the precise design procedures and steps are provided. Designing experiments and analysing the results are covered in the fourth chapter. This section mainly explains how well the system works and analyses the feedback evaluation results. The final chapter is the conclusion. The research findings are outlined in this chapter, along with an explanation of the study's limitations and possible future research directions.

## 2. Related Work

Schools are paying increasingly more attention to music instruction as a crucial component of high-quality education. Music education is being gradually incorporated into education as it rapidly develops digitally and informatically. A system that uses computers to support education is known as a computer-assisted education system. Many academics have currently conducted pertinent research on the teaching assistant system.

Yuan et al. developed a demand analysis for the digital classroom teaching assistance system based on the actual circumstances of classroom instruction in schools and made an overall design of the system based on those circumstances [9]. A method of outlier detection based on clustering and density was proposed by Huang. The local outlier detection algorithm was used after K-means clustering and pruning, greatly reducing algorithm complexity [10]. Through their research on evaluating the effectiveness of classroom instruction, Wang and Mu suggested that the use of machine learning for evaluating the effectiveness of classroom instruction can significantly increase evaluation efficiency and streamline the evaluation process [11]. The implementation of a rule-based uncertainty expert system was examined by Gong et al., who also proposed a general implementation plan for an AI-based assisted teaching system [12]. Expert systems, according to Bian, serve an explanatory purpose. While it is running, it can respond to queries from users and explain how issues are resolved as well as the conclusions reached at the end of the process. Users can understand the reasoning process and have more faith in the expert system because the explanation process is transparent [13]. The fundamental requirements for the digital music classroom teaching assistant system are presented by Gooch et al., followed by a division of the system into three modules and a detailed explanation of the functions of each module [14]. In order to increase the precision of the indicators used to measure teaching quality, Boulay proposed a mathematical model of teaching quality evaluation based on wavelet NN (neural network). However, there are drawbacks to using NN, including how simple it is to fall into local extreme points and how strongly sample-dependent it is [15]. The calculation rules and inference rules of probability are the main subjects of the discussion in He et al. By introducing a membership function, possibility theory can calculate uncertainty in terms of likelihood [16]. A teaching assistant expert system with good interactivity and a user-friendly interface for resource sharing, Jin emphasises “strengthening students' autonomous learning ability” and uses the technical background of AI [17]. It has developed into a potent teaching aid for teachers.

This study combines education and teaching theory with machine learning methodology to design and implement a music teaching assistant system, that is, in line with the actual teaching situation. It is based on an in-depth analysis of related literature. In this paper, the system requirements, as well as the application of software engineering, computer networks, Website architecture, and other knowledge-related topics, were analysed. On the basis of this analysis, the system's overall structure and its internal modules were designed in a somewhat detailed manner. The system is split into learning modules for music fundamental theory, music common sense, music appreciation, and evaluation management. Online learning can provide mining potential and increase the effectiveness of critical information tools thanks to JSP practical technology that has been optimised for practical use and Oracle database data intelligent retrieval for music teaching work. For each functional module, test cases are created and executed. The study demonstrates the system's good portability and scalability, as well as its straightforward, effective algorithm and user-friendly interface. This study is a valuable resource and aid for music educators.

## 3. Methodology

### 3.1. CAI

CAI is the use of computers to replace teachers in teaching, the teaching content in a variety of courseware can enable learners to choose different content for learning according to their own situation [18]. Computer-aided system is mainly composed of three parts, which are computer hardware, system software, and course software. The auxiliary teaching system replaces the single teaching mode of the conventional music lesson from the past and can offer students a rich, colourful, three-dimensional interactive teaching interface with images and texts, audio, and video, making it simple to pique their interest in learning. It can diversify and visualise the teaching material, making it easier to teach students according to their aptitude. The effectiveness and calibre of music education can be raised by making full use of CAI to investigate new educational models and by integrating computer and Internet information technology into music teaching activities. Projector, curtain, exhibition stand, control computer, active sound box, etc., are some of the major components of computer hardware. The most crucial component of a computer-aided system is computer hardware. One could say that the main advancement of the CAI system has a crucial relationship with the advancement of computer hardware. Hardware for computers is thus the cornerstone of the entire CAI. The teaching philosophy, approach, and content can all be expressed as knowledge in CAI. One of its key technologies is the way to deal with the issue of the formal expression of knowledge as well as the access and call of knowledge. The knowledge base can generally be used as the environment in which intelligent CAI is built [19]. Production representation is used in the expert-aided teaching system to express rules. Mechanical learning, guided learning, inductive learning, analogy learning, and explanation-based learning are a few examples of machine learning techniques. This is a brand-new teaching strategy that has emerged recently. A teaching-type expert system's job is to instruct and coach students using the best teaching strategy and method based on their traits, weaknesses, and foundational knowledge [20]. The interface between knowledge engineers, domain experts, and expert systems is the knowledge acquisition organisation. The knowledge is added to the knowledge base through interaction with domain experts and knowledge engineers, creating a good performance knowledge base that can be continuously updated and supplemented.

The system software of CAI mainly includes an operating system, language processing system, various tool software, writing system, etc. Among them, the system software is an important part of the entire CAI, it can provide word processing, animation, video recording, courseware generation, and other functions for the classroom and students to provide convenience. For example, using the PowerPoint programme, a teacher can play a variety of course materials in the form of slides and animation, which will help students better understand and master the necessary key knowledge. The knowledge base serves as the basis for knowledge reasoning and expert systems. Knowledge about teaching materials and other topics can be expressed with facts and regulations in the knowledge base and stored there. The process of reasoning from the knowledge base and ultimately obtaining the desired outcomes is the process of teaching and learning. The database is used to store the system's pertinent data, including user-inputted data used to operate the system, intermediate reasoning results, and output results after the issue have been resolved. The initial facts supplied by the user are stored at the start of the problem-solving process, and the conclusions of each step of the reasoning process are also stored in the database. In general, the course software of CAI is the teaching application software, that is, written in accordance with the requests of the teachers or the course requests of each school. CAI currently has access to software that can create course materials automatically. Teachers can directly generate the desired courseware through the system, relieving them of the burden of creating courseware with diagrams and voiceovers. The CAI offers a place where students can take advantage of their opportunities for music practise and develop their ability to compose music. In order to help students develop their musical perception, memory, imagination, thinking, and other skills, CAI can offer them a broad range of music knowledge and information, that is, aligned with the qualities of artistic associative thinking and memory. It can also encourage students' aesthetic feelings and creative ability.  Figure 1 depicts the system architecture of this pap.

The man-machine interface component of the CAI is merely a user interface. Its implementation can be complex or take on a variety of shapes [21]. Human-machine interfaces need to understand natural language because people want to be able to converse with machines like human experts rather than just using simple commands. The primary purpose of a computer-aided education system is to support teachers in their instruction of students in a classroom setting. (1) It can assist teachers in teaching students according to their aptitude. (2) It can fully exploit the active role of the students, who are engaged in active rather than passive learning. (3) It can conserve educational resources, make learning convenient for students, and provide high-quality education to a broad audience. At the same time, computer-aided education system also has some disadvantages, such as: (1) Large investment in equipment; moreover, there are risks that the system updates too quickly and the equipment cannot meet the needs of subsequent updates. (2) The level of intelligence and popularization of CAI system is limited, and it cannot completely replace teachers. (3) There may be a problem that the developed systems and products can not really meet the needs of education. For an expert system, its performance convenience, effectiveness, reliability, and maintainability can be considered from many aspects. Convenience refers to the degree of convenience provided by the expert system for users. Effectiveness refers to the time cost and complexity of the problem solved, the representation of knowledge, and the method or organisation of using knowledge when the system actually solves the problem. Reliability refers to the reliability of the answers provided by the system to the users and the stability of the system. Maintainability refers to whether the expert system is convenient for modification, expansion, and improvement. Up to now, the vast majority of traditional CAI have preset all teaching information in courseware by programming. Once such CAI courseware is made, any teaching changes will bring great inconvenience to the maintenance work. Therefore, the existing CAI system faces many challenges.

### 3.2. Construction of Music Teaching Assistant System Based on Machine Learning

The purpose of this paper is to develop a piece of music teaching assistant programme to support teachers' in-class instruction by examining the features of the current music classroom environment and employing the most up-to-date computer technology to do so [22]. This paper designs the system based on Web service architecture in accordance with the development trend of Web service architecture to realise music-assisted instruction system and all possible new requirements. Including modules for user management, evaluation management, music appreciation, learning about music, etc. The development of the music teaching assistant system should adhere to the steps and principles of software engineering, including the five stages of requirement analysis, system design, system realisation, test, and maintenance, just like other large-scale software development processes. The entire auxiliary teaching system consists of the learning modules for music fundamental theory, music common sense, music appreciation, evaluation management, and user management. Knowledge must be expressed in a specific way that computers can understand in order to make machines intelligent. It is true that knowledge representation has a direct impact on how well an expert system performs. This article's knowledge base is used to store domain knowledge, which is separate from other system components and contains a substantial amount of facts and rules in all the problem domains that need to be solved. The following traits should, in general, be present in a good knowledge representation: (1) Knowledge should be easy to modify and expand thanks to the knowledge representation. (2) The aforementioned method ought to be straightforward and simple to comprehend. (3) The method should be explicit and clear.  Figure 2 displays the expert system's fundamental architecture as well as the network topology diagram for the system.

It is crucial to assess the performance and quality of computer software by looking at how simple and intuitive the user interface is to use. The software requirement analysis, basic design, and system test phases of the design and development process are all involved in the user interface design. For users to spend less time learning how to use the system and to start using it more immediately, it should have a unified user interface and operation mode. Extensible application markup language, which is discussed in this paper, allows you to create rich interface styles and templates as well as quickly define and layout interface elements, making it possible to create an interface, that is, both beautiful and atmospheric. The interface of the music teaching assistant system uses the humanised design approach and includes a variety of remarks, explanations, and help, making it simple for network users to accept and use. The system can successfully finish the fundamental operation process upon the first login. The interface's network links and function buttons make sense, and the links' and buttons' names are simple to decipher. The rules of music are complicated and flexible, whereas they are more random in the music classroom. The method of combining NN with an expert systems is thus used in this paper to increase the system diagnosis' accuracy and personalization. Make logical and intuitive thoughts complementary to one another. In this study, the diagnostic process realises the nonlinear mapping of input and output, and the final diagnosis result is obtained by using NN. This transformation of the empirical knowledge of music experts into a nonlinear problem allows for the realisation of the nonlinear mapping of input and output. The minimum mean square error learning approach is used by BPNNs (back propagation neural networks). Errors are reversely propagated to the input layer during the learning phase, and input vectors are forwarded to the output layer by layer during the working phase. The output layer in the three-layer BPNN algorithm consists of

(1) $$\begin{array}{c} o_{k}=f\left({\text{net}}_{k}\right),\;k=1,2,3,\ldots ,l,\\ {\text{net}}_{k}=\sum_{j=0}^{m}w_{jk}y_{j},\;k=1,2,3,\ldots ,l. \end{array}$$

For hidden layers, there are:

(2) $$\begin{array}{c} y_{j}=f\left({\text{net}}_{j}\right),\;j=1,2,3,\ldots ,m,\\ {\text{net}}_{j}=\sum_{i=0}^{n}v_{ij}x_{i},\;j=1,2,3,\ldots ,m. \end{array}$$

The transfer functions *f*(*x*) are all unipolar Sigmoidal functions:

(3) $$\begin{array}{c} f\left(x\right)=\frac{1}{1+e^{-x}}. \end{array}$$

It has the characteristics of continuous and derivation and:

(4) $$\begin{array}{c} f\left(x\right)=f\left(x\right)\left[1-f\left(x\right)\right]. \end{array}$$

The function of each neuron is the sigmoid function, and the output nodes are:

(5) $$\begin{array}{c} y_{t}=F\left(S_{t}\right)=F\left[\sum_{i=1}^{k}w_{it}h_{it}h_{i}-\theta_{i}\right]t=1,2,3,\ldots ,l. \end{array}$$

For hidden layer nodes:

(6) $$\begin{array}{c} h_{i}=F\left(S_{i}\right)=F\left[\sum_{j=1}^{m}w_{ji}x_{j}-h_{j}\right]i=1,2,3,\ldots ,k. \end{array}$$

Since the system consists of multiple modules, each of which also has a number of functions, the overall design of the system is carried out in order to smoothly achieve coordinated operation between the system's modules and its overall function while ensuring the system's stability and future function expansion. The B/S three-layer architecture is the primary design choice for the modern information technology-based music assistant teaching system. Network layer, application layer, and data layer are the three levels that make up this hierarchy. B/S mode offers the benefits of low software deployment costs, simple network access, quick network application upgrades, and quick system maintenance. In this structure, the user interface is entirely realised through the WWW browser, and the B/S mechanism realises the original powerful functions that call for difficult special software to realise by utilising the continuously developed and well-liked browser technology, thus saving the development cost. The database server should have enough resources for data backup and data recovery, and the Web application server is configured for a large number of levels of network applications in high bandwidth, load-balancing manner. When designing the system flow, this paper follows the principle of reducing the complexity of the system as much as possible, and simplifies the flow step by step to remove unnecessary intermediate links; try to keep the process as simple as possible. Of course, the process is not as simple as possible, and the bottom line must be to ensure the integrity of the function. The whole system includes four users: domain experts, music teachers, students, and system administrators. When a user logs in, the user has different module operation permissions according to different identities. Based on the actual teaching situation, the design and implementation of this system should maximize the promotion of system professionalism, in ensuring the accuracy of the case, and improve the quality of the system.

The knowledge base rules in this system are founded on credibility. As a result, the machine for uncertainty reasoning is implemented. Create the following fuzzy relationship:

(7) $$\begin{array}{c} \mu_{z}=\left\{\mu_{y}\cdot W\right\}. \end{array}$$

Among them, *μ*_*z*_ is the conclusion vector, and · is the logical operator. Solve to get the reasoning mode of this system:

(8) $$\begin{array}{c} \mu_{y}⟶\mu_{CF}⟶\mu_{z}. \end{array}$$

Among them, *μ*_*y*_ represents the vector of the forward reasoning conclusion *y* quantized, namely:

(9) $$\begin{array}{c} {\left[\mu_{y_{1}},\mu_{y_{2}},\mu_{y_{3}}\ldots ,\mu_{y_{n}}\right]}^{T}, \end{array}$$

*W* is the weight vector [*w*_1_, *w*_2_, *w*_3_,…, *w*_*n*_]. Order:

(10) $$\begin{array}{c} \mu_{p}=\mu_{y}\cdot W. \end{array}$$

Assuming that *μ*_*p*_ is a weighted logical formula, then:

(11) $$\begin{array}{c} \mu_{p}=\sum_{t=1}^{n}w_{i}\cdot \mu_{y}. \end{array}$$

The truth of this conjunction is the weighted cumulative sum of the truth of each subitem. Therefore, the truth degree of the whole equation increases with the increase of the true degree of each sub-equation.

Entity, attribute, and connection are the three main components of the database E-R graph, which is a set model of the relational schema of relational database results. Therefore, the process of transforming three components into a relational model is the essence of turning an E-R graph into one, in accordance with the top-down analysis method's specifications. Separating hierarchical modules can do two things: on the one hand, it can make the system's structure explicit and clear, making it easier to understand the division of labour during the development phase; and on the other hand, it can make the system simpler to expand and maintain. Keep the low coupling and high cohesion between the system modules when splitting them up. So that all clients can be connected to the middle layer through the controller, and so that the middle layer can then realise interaction with the database, the business rules, logic, mapping, data access, and other work can be placed in the middle layer to deal with. The edited score, including the pre-performance function of the score and the saving function of the score, is the focus of the score preview and saving sub-module in this paper. The ability to preview an edited music score in real time, identify errors as they arise, and make corrections makes it much easier for music teachers to teach in the classroom. Giving full play to the role of the “music teaching auxiliary system” in the learning field of musicology can activate the online learners' desire for performance and creative impulse, and show their personality and creative ability in the interactive participation so that their imagination and creative thinking can be given full play.

## 4. Result Analysis and Discussion

The auxiliary system for music instruction in the preceding chapter is built in this essay. This chapter tests each system module to confirm the functionality of the created music teaching assistant system and algorithm. System testing and analysis is a difficult and complex task. Numerous Web-based applications with their practical, quick, user-friendly, and other qualities continue to be the focus of software development due to the rapid advancement of network technology. This study tests and evaluates complex systems using various techniques and methods from traditional software testing. The distinctiveness and complexity of Web application systems also present greater testing requirements. Hardware and software for PCs are required for the music teaching assistant system test to function properly. Utilizing the Windows operating system is tested in this chapter. The simulation module is used to provide the function simulation of the modules directly under the main module, ensuring that each module can function normally. The main module of the system serves as the main body of the test.  Table 1 displays the results of us login test.

The experimental results in the table show that the system can run normally and meet the corresponding performance requirements. The functions provided by the system are consistent with the original design, and the system can meet the needs of actual use. Real-time is also one of the important design principles of the music teaching assistant system. The real-time performance here mainly means that the results of user operations should be responded to within a time that does not affect the system function and effect. In this paper, we test the real-time performance of the system. The experimental results are shown in Figure 3.

Figure 3 illustrates the high real-time performance of the system used in this paper. Nevertheless, stability is crucial for any software or system, and it can significantly enhance user experience. The stability of various systems will therefore be tested in the following step, and the results will be compared and analyzed. The teaching of music is less mandatory than the teaching of other subjects. The rules of music are also intricate and subject to change. This necessitates extremely high fault tolerance and stability from the music teaching assistant system. Therefore, to ensure the stability of the system, we should fully consider all potential scenarios when designing the auxiliary system for digital music classroom teaching.  Figure 4 displays the outcomes of various systems' stability tests.

The stability of the system in this paper can reach 93.87%, which is higher than the traditional teaching system's 9.14%, as can be seen from Figure 4. As a result, the system in this paper has better stability and can satisfy actual needs.  Figure 5 displays the outcomes of the safety tests conducted on various systems.

It can be seen from the result analysis that the system in this paper has high security. In this paper, a variety of enhanced key algorithms and network security license files to improve the security of network data and deep-level protection of the database, and the use of new technologies to encrypt the data storage database. In order to test the actual use effect of the system, 100 users were invited to rate the use of system. A 5-point scale is used for scoring; A larger value gives a higher score. The user's rating is shown in Table 2.

By contrast, the interface of this system is friendly and has a certain aesthetic feeling. And the operation is convenient and the professionalism is strong. Which can meet the user's aesthetic and practical teaching application needs. In this chapter, the algorithm is tested on the Scikit-learn platform using the Iris data set, and the result of the algorithm's accuracy is shown in Figure 6.

The test results demonstrate that the proposed algorithm has the highest accuracy, which can exceed 90% in small sample data sets. The algorithm presented in this paper can significantly reduce the amount of data preprocessing work required and enable the model's accuracy to reach its maximum performance even with sparse data. The results of comparing the students' test scores before and after using the music teaching aid system in this paper are displayed in Figure 7.

According to the analysis of the data in Figure 7, the student's scores increased as a result of the use of this method to help with teaching management. The outcomes demonstrate the viability and effectiveness of the methodology used in this paper. This chapter uses the Iris dataset to test the algorithm on the Scikit-learn platform and tests each module of the built-in music teaching assistant system in order to validate its effectiveness. The stability of the music teaching assistant system developed in this paper can reach 93.87%, which is higher than the traditional teaching system's 9.14%. Additionally, the system's user satisfaction can reach 92.16%, according to the results of numerous experiments. This outcome demonstrates that the system performs admirably and satisfies the user's requirements for the teaching application's practicality and aesthetic appeal. It checks the system's entire functionality and guarantees that each functional module is operating normally.

## 5. Conclusions

There are numerous machine learning model creation techniques; the model chosen for the current problem should be combined with the problem's actual context. Following a comparison and analysis of the well-known music teaching assistant system, we develop a machine learning-based music teaching assistant system and select the most appropriate computer technology to implement it in accordance with the system's requirements. We introduce a diversity measure to ensure that the base learner has good diversity in order to enhance the algorithm's performance. Utilizing the Iris data set, the algorithm was tested on the Scikit-learn platform. Tests reveal that even with little data, the proposed algorithm can produce results with high accuracy. The stability of the music teaching assistant system developed in this paper can reach 93.87%, which is higher than the traditional teaching system's 9.14%. Additionally, user satisfaction with the system can reach 92.16%, according to the results of numerous experiments. This result demonstrates that the system performs at a high level and satisfies the user's requirements for both the teaching application's aesthetic appeal and practicality. It has some theoretical and practical importance for the field of teaching aids, as well as some reference value for pertinent researchers. Although this paper has produced some research findings, many other factors were not taken into account during the design phase due to time constraints and my level of expertise. In the future, work will also be done to improve the music teaching auxiliary system and expand its functionality, while also taking into account the system's unique needs.

## Figures and Tables

**Figure 1:** System architecture diagram of this paper.

**Figure 2:** Basic structure and network topology diagram of an expert system.

**Figure 3:** Real-time test results of the system.

**Figure 4:** Stability test results for different systems.

**Figure 5:** Safety test results for different systems.

**Figure 6:** Accuracy results of the algorithm.

**Figure 7:** Student achievement comparison result.

**Table 1:** User login test table.

User ID	Test user001	
Functional description	System functions	
Experimental purpose	Test the system for proper use	
Precondition	Enter the web address to enter the system login interface	
Inputs/actions	Desired output/response	The actual situation
Open login page	Page complete, each function button in the operable state	As expected
Input required is not filled in	System prompt required	As expected
Do not enter the password, only enter the user name, click the login button	The system prompts the user to fill in the user's name and password information	As expected
Just enter the password, do not enter the user's name, and click the login button	The system prompts the user to fill in the user's name and password information	As expected
Enter the correct user ID and password	The system prompts login success, page jump	As expected
No attachments were selected for uploading the lecture video	The system prompts that the attachment content cannot be empty	As expected
Attachment too large	System attachment is too large, suggest ftp upload or web share	As expected
Attachment upload timed out	The system prompt timed out, please upload again	As expected
Drag the progress bar on the video playback page	The video playback progress advances or retreats to the designated bit accordingly	As expected
Click the content editor ribbon	Ribbon function is used normally	As expected
Enter matches	The system prompts that the operation was successful	As expected

**Table 2:** User's subjective scoring scale.

System	Interface friendliness	Ease of use	Professionality	Satisfaction (%)
Traditional auxiliary teaching system	3.12	3.25	2.19	78.97
NN-based auxiliary teaching system	3.26	3.34	3.59	83.02
AI-based auxiliary teaching system	4.11	3.28	4.29	91.48
This article auxiliary teaching system	4.52	4.37	4.48	92.16

## Data Availability

The data used to support the findings of this study are available from the author upon request.

## References

[1] Otchere E. D. (2015). Music teaching and the process of enculturation: a cultural dilemma. *British Journal of Music Education*.

[2] Ho T. K. L., Lin H. S., Chen C. K., Tsai J. L. (2015). Development of a computer-based visualised quantitative learning system for playing violin vibrato. *British Journal of Educational Technology*.

[3] Liikkanen L. A., Aman P. (2015). Shuffling services: current trends in interacting with digital music. *Interacting with Computers*.

[4] White R. (2020). Authentic learning in senior secondary music pedagogy: an examination of teaching practice in high-achieving school music programmes. *British Journal of Music Education*.

[5] Iliaki G., Velentzas A., Michailidi E., Stavrou D (2019). Exploring the music: a teaching-learning sequence about sound in authentic settings. *Research in Science & Technological Education*.

[6] Han X. U. (2015). *Learning Field Curriculum of Germany:Transformation of Teaching System of Vocational Education*.

[7] Tan R. A., Alpert P. T. (2013). A teaching intervention to improve the self-efficacy of internationally educated nurses. *The Journal of Continuing Education in Nursing*.

[8] Gong Z. (2017). Research on multimedia instruction and music flipped classroom teaching model under internet background. *Boletin Tecnico/Technical Bulletin*.

[9] Yuan Y., Ni X., Cao Y. (2020). A magnetic electrode modified with hemoglobin for determination of hydrogen peroxide: distinctly improved response by applying a magnetic field. *Mikrochimica Acta*.

[10] Huang W. (2021). Simulation of English teaching quality evaluation model based on Gaussian process machine learning. *Journal of Intelligent and Fuzzy Systems*.

[11] Wang S., Mu M. (2021). Exploring online intelligent teaching method with machine learning and SVM algorithm. *Neural Computing & Applications*.

[12] Gong W., Tong L., Huang W., Wang S (2018). The optimization of intelligent long-distance multimedia sports teaching system for IOT. *Cognitive Systems Research*.

[13] Bian H. X. (2016). Application of virtual reality in music teaching system. *International Journal of Emerging Technologies in Learning*.

[14] Gooch D., Benton L., Khaled R., Lukes D., Vasalou A (2016). Creating bridges: the role of exploratory design research in an intelligent tutoring system project. *Interacting with Computers*.

[15] Boulay B. D. (2016). Artificial intelligence as an effective classroom Assistant. *IEEE Intelligent Systems*.

[16] He H., Yan H., Liu W. (2020). Intelligent teaching ability of contemporary college talents based on BP neural network and fuzzy mathematical model. *Journal of Intelligent and Fuzzy Systems*.

[17] Jin C. (2017). Analysis of music teaching mode innovation based on intelligent classroom and multimedia system. *Revista de la Facultad de Ingenieria*.

[18] Li Y., Xu J., Liu L. (2017). Post-stroke unilateral spatial neglect treated with acupuncture and rehabilitation: a randomized controlled trial. *Revista de la Facultad de Ingenieria*.

[19] Zhang J., Feng H. (2021). Mobile terminal system of intelligent college English teaching and training mode. *Mobile Information Systems*.

[20] Borges J. A., Tome D. (2014). Teaching music to blind children: new strategies for teaching through interactive use of musibraille software. *Procedia Computer Science*.

[21] Kim E. (2013). Music technology-mediated teaching and learning approach for music education: a case study from an elementary school in South Korea. *International Journal of Music Education*.

[22] Wen X. (2020). Using deep learning approach and IoT architecture to build the intelligent music recommendation system. *Soft Computing*.

